The article "A novel industrial-scale strategy to prevent degradation and caking of ammonium nitrate" was published in 2020. Journal: Heliyon.

# A novel industrial-scale strategy to prevent degradation and caking of ammonium nitrate

**DOI:** 10.1016/j.heliyon.2020.e03628

**Published:** 2020-03-25

**Authors:** Ahmet Ozan Gezerman

**Affiliations:** Yildiz Technical University, Department of Chemical Engineering, Istanbul, Turkey

**Keywords:** Chemical engineering, Nitrogenous fertiliser, Sodium silicate, Silicic acid, Calcium lignosulfonate

## Abstract

Several research studies have been performed to minimise the hygroscopicity of ammonium nitrate for increasing its commercial value and decreasing the nitrogen content. In this study, the hygroscopicity of ammonium nitrate was reduced using silicic acid, calcium lignosulfonate, and sodium silicate in the two-stage vacuum ammonium nitrate production process. Degradation of ammonium nitrate was observed after two years of storage, which is considered a standard by the European Fertilizer Manufacturers Association.

## 1 Introduction

Ammonium nitrate is the chemical fertilizer most preferred by consumers because of its effectiveness in the agricultural industry [1]. During the transfer of ammonium nitrate and before it reaches the consumer, various quality problems such as caking, and degradation are encountered [2]. Commercially, ammonium nitrate containing 26% and 33% nitrogen is manufactured in the production process [1]. To obtain this nitrogen concentration, ammonium nitrate is diluted with calcium carbonate (ground to a maximum particle size of 150 μm) and dolomite [3]. With the addition of such chemicals, the physicochemical properties of ammonium nitrate, such as hygroscopicity, are influenced in various ways via the creation of new and undesired chemical species [4]. It is very important to mitigate the hygroscopicity of ammonium nitrate to maintain the desired nitrogen content of ammonium nitrate and prevent degradation of the fertiliser under the given storage conditions [5]. To prevent the degradation of ammonium nitrate, several alternative additives have been tested. In this regard, calcium trialkylamine, potassium dimethyloctylamine, dimethyl decylamine, and dimethyl laurylamine have been successfully used [6].

Another process to prevent the degradation of the ammonium nitrate fertilizer is by coating it with a mixture of 10–50% wax and 40–90% mineral oil. The chemical coating consists of high molecular weight polyisobutylene. It has been reported that this process substantially limits the water absorption and dust formation properties of the ammonium nitrate fertilizer [7].

In another study on mixtures of ammonium nitrate and ammonium sulfate, the thermal stability of ammonium nitrate was investigated, the nitrogen concentration in ammonium nitrate decreased to 21%, and the caking tendency decreased [8]. In yet another study to reduce the hygroscopicity of ammonium nitrate, polyethylene- or polypropylene-based polymer material was mixed with a wax-based material to form the protective layer for fertilizer granules. However, the use of hydrophobic polyethylene was restricted by its insolubility in water [9].

The article "A novel industrial-scale strategy to prevent degradation and caking of ammonium nitrate" was published in 2020. Journal: Heliyon.

In another study, the surface properties of ammonium nitrate were improved by coating it with polyvinyl acetate (PVAC), wax, and polyethylene glycol (PEG) [10].

A different study also found that adding 26–34% urea and 1–15% elemental sulfur limits the moisture absorption properties of ammonium nitrate and significantly reduces its degradation [11].

It has been found that the addition of 0.25–5.0% tripotassium phosphate to the production process reduces the moisture absorption properties of ammonium nitrate, thereby decreasing the tendency towards aggregation [12].

Chemical additives such as sodium alkyl sulfate, potassium alkyl sulfate, monoethanolammonium alkyl sulfate, diethanolammonium alkyl sulfate, and triethanolammonium alkyl sulfate have been studied to limit the moisture absorption properties of nitrogenous fertilizers such as ammonium nitrate; positive results have been reported [13].

In another study on anti-caking in nitrogenous fertilizers, it was found that moisture absorption properties were limited by coating them with 20% bitumen [14].

Another chemical agent that is added to the process of producing ammonium nitrate fertilizer to resolve the issue of caking is a mixture of 30–90% phosphoric ester and 70–10% fatty trialkylamine. This additive improves the surface properties of ammonium nitrate [15].

Another study substantially limited the moisture absorbing properties of ammonium nitrate by adding a 5% citric acid solution to the polysaccharide sugar solution to the process of producing ammonium nitrate [16].

Another method proposed as a way to reduce the moisture absorption of fertilizers is covering the fertilizer surface with a vacuum tower asphalt extender (VTAE) [17].

The surface properties of ammonium nitrate particles were also greatly improved by the use of an inorganic coating containing 8–25% ammonium sulfate [18].

Alumina (Al_2_O_3_) added to the ammonium nitrate solution in concentrations from 0.01 wt% to 2 wt% substantially limits the tendency of the latter to absorb moisture [19].

Other salts such as superphosphate and ground rock phosphate have been added to prevent the degradation of ammonium nitrate, and the maximum salt concentration in the ammonium nitrate solution was 40% [20].

To prevent the degradation of ammonium nitrate, various additives such as sodium silicate and silicic acid were used, which imparted non-caking properties during the storage duration of two years [1]. The effects of sodium sulfate on the degradation of ammonium nitrate were investigated, and it was reported to result in a long storage life for ammonium nitrate [21]. The hygroscopic properties of ammonium nitrate were improved by coating urea on its surface. In this case, the porous structure of ammonium nitrate was filled with urea, and a film that limited the hygroscopic properties of ammonium nitrate was formed [22]. The effects of crystal structure on the degradation and caking problem were reported, and the phase changes of ammonium nitrate at different temperatures were investigated [23].

The article "A novel industrial-scale strategy to prevent degradation and caking of ammonium nitrate" was published in 2020. Journal: Heliyon.

In this study, ammonium nitrate was produced via a two-stage process by using nitric acid (55%) and anhydrous ammonia (99.9%), as condoned by the European Fertilizer Manufacturers Association (EFMA), and sodium silicate was added for diluting ammonium nitrate. Sulfuric acid is used to minimise the production of carbon dioxide during ammonium nitrate. However, the sulfate ions react with the nitrate ions in nitric acid, leading to the formation of a double salt. Silicic acid added in the ammonium nitrate dilution stage eliminates sulfate ions and prevents the formation of double salts.

The surface of prilled ammonium nitrate was then coated with calcium lignosulfonate and over two years of storage, no caking and degradation of ammonium nitrate was observed. All processes were investigated by instrumental analysis such as scanning electron microscopy (SEM), ion chromatography, and XRD diffraction analysis.

The following materials were used in the ammonium nitrate production: nitric acid (55%); anhydrous ammonia (99.9%); pure silicic acid (1 mL/5.6 mL sulfuric acid); 600 ppm sulfuric acid 98% wt; 12.5% pure sodium silicate, and 12.5% pure calcium carbonate. All chemical materials in this study were supplied by Merck (Istanbul, Turkey).

Sodium silicate is added in the presence of calcium carbonate to dilute ammonium nitrate, with the aim of monitoring the cooling rate of ammonium nitrate that solidifies during cooling, and to reduce its pore size. However, the aim was to determine the optimum concentration of both sodium silicate and calcium carbonate that could be added.

Nitrogenous fertilizers are vital to yield yields from agricultural areas. Therefore, the production of nitrogen fertilizers is important in terms of meeting the need. Fertilizer introduced into the soil must meet certain quality parameters. However, due to the high moisture absorption feature of ammonium nitrate, it is not always possible for fertilizers to provide quality parameters. In order to prevent this problem, researchers have been going through method research for a long time, but the solutions offered do not meet the long storage period. In this study, in order to meet this long storage period (2 years), various chemical additions have been made and it has been achieved that the final product provides fertilizer specifications.

The article "A novel industrial-scale strategy to prevent degradation and caking of ammonium nitrate" was published in 2020. Journal: Heliyon.

Most of the studies reported in the literature have not been able to prevent changes in the physical and chemical structure for the 2-year time period, which is accepted by EFMA as a standard for the quality of fertilizers. In the studies carried out, the degradation in the structure of ammonium nitrate occurred together with the humidity of the air in the period after 6 months. In addition, the studies reported in the literature are laboratory-scale and did not create long-term effects due to the lack of economic concerns. Along with the chemical additives recommended in the process here, a 2-year storage life has been successfully achieved in accordance with EFMA standards.

## 2 Materials and methods

In this study, the preferred method for industrial ammonium nitrate production is the two-stage vacuum method [10]. In the two-stage ammonium nitrate production, liquid ammonia (5 °C, 9 kg/cm^2^) is vaporised or conditioned (15 °C, 6.1 kg/cm^2^) in an evaporator (Table 1). After that, ammonia is reacted with nitric acid in a pipe-type reactor to obtain 80% ammonium nitrate, which is concentrated to 94% in a first-stage vacuum evaporator and to 99.7% in a second-stage vacuum evaporator. After the ammonium nitrate solution reaches a concentration of 99.7%, calcium carbonate is added for dilution to obtain 26% and 33% nitrogen-containing ammonium nitrate. Calcium carbonate forms CO_2_ gas in the ammonium nitrate reaction ambience, decreasing the viscosity of ammonium nitrate. Hence, cracking occurs on the surface of ammonium nitrate during prilling, and foaming occurs in the ammonium nitrate dilution process. For decreasing the foaming problem, sulfuric acid (98% w/w) is added to the ammonium nitrate dilution ambience. The amount of sulfuric acid added is found to be 600 ppm. The addition of sulfuric acid creates crystal bridges, which may lead to caking with nitrate salts in ammonium nitrate under the storage conditions. To eliminate double salts sourced by sulfuric acid, silicic acid is added to the reaction ambience (1 mL silicic acid/5.6 mL sulfuric acid) (Figure 1). The final ammonium nitrate product is prilled by cooling in a prilling tower.

**Table 1:** Pressure and temperature values in the production process [24].

Stage	Pressure/kg cm^−2^	Temperature/°C
Ammonia evaporation	6.1	15
Ammonium nitrate production reactor	5.6	125
I. stage evaporation	3	125
II. stage evaporation	3	175
dilution with filler as CaCO_3_	1	175
prilling	1	175

The article "A novel industrial-scale strategy to prevent degradation and caking of ammonium nitrate" was published in 2020. Journal: Heliyon.

**Figure 1:** Two-stage vacuum ammonium nitrate production process.

The equipment used in the ammonium nitrate production process completed in this study included: an ammonia evaporator which was used for bringing ammonia to reaction condition (15 °C); a reactor to contain the reaction between nitric acid and ammonia; a solution tank for storage of 80% ammonium nitrate after reaction; stage evaporators for concentrating the ammonium nitrate produced; a solution tank for adding CaCO_3_ and sodium silicate to the ammonium nitrate concentrated in evaporators; a prilling bucket for ammonium nitrate produced, and a rotating drum coated with an anticaking agent to contain the prilled ammonium nitrate.

### 2.1 Electron microscopy analysis

Electron microscopy analysis reveals the morphological structure of prilled ammonium nitrate. For this purpose, a Carl Zeiss DSM-960A system was used and an analysis was performed according to the ASTM E986-97 standard. To better understand the surface properties of ammonium nitrate, the following conditions were used: accelerating voltage, 1–30 kV; useful magnification, 10–30000×; resolution, 70 Å.

### 2.2 Ion chromatography analysis

For analysing the amount of double salts in ammonium nitrate, the amounts of nitrogen and other ions (anion-cation) were analysed by ion chromatography according to the ASTM E1151-93 standard by using a Shimadzu Prominence HIC–NSn system. The working parameters were as follows: 0.01–51200 μS/cm; flow rate, 0.001–5 mL/min.

### 2.3 Screen sieve analysis

Ammonium nitrate solution that is diluted to the desired concentration by using additives is prilled in a prilling bucket. According to commercial requirements or as per the universal standard, the average particle size of prilled ammonium nitrate should be 2 mm, which is achieved when using a conical prilling bucket. The rotating speed of the bucket can also affect the particle size. A Vibratory Sieve Shaker AS 200 was used, and the analysis was performed by employing the method prescribed by ASTM E11-09 [1].

The sieve vibration machine (manufactured by Retsch, Germany) operates in the vibration width between 0–3.0 mm and 100 g of weighed sample is sieved for 5 min by vibrating from the stacked sieves for analysis with 6 particle sizes (3.35, 2.5, 2.0, 1.0, 0.5 and under sieve) [1].

The percentage of retained material is calculated simply by:

(1) T,%=(M1M)×100

where T is the percentage of retained material on a sieve (%), ${\text{M}}_{1}$ is the sample mass under the sieve, g: is the total sample mass, g.

The article "A novel industrial-scale strategy to prevent degradation and caking of ammonium nitrate" was published in 2020. Journal: Heliyon.

### 2.4 Crushing strength analysis

Crushing strength is the maximum compressive load at which 2 mm fertiliser granule is broken completely. A crushing strength testing machine, Instron Test System (Model 4411) was used.

### 2.5 Analysis of sulfate

During ammonium nitrate production, sulfate ions form a double salt with the nitrate, and this leads to caking because of the creation of crystal bridges. Therefore, excess sulfate should be removed by the precipitation of barium sulfate using diluted HCl (d20 = 1.18 g/mL), BaSO_4_ solution (122 g/L), and AgNO_3_ solution (5 g/L). Analysis samples were prepared by mixing HCl (20 mL) and H_2_SO_4_ (50 mL), which was diluted to 300 mL with demineralized water and boiled, followed by the slow addition of barium chloride (20 mg) and boiling for a few minutes. This hot solution was allowed to stand for 1 h. When the solution became completely clear, it was filtered, and the precipitation obtained was washed with silver nitrate until the chloride ions were completely removed. The filter paper and precipitate in porcelain crucible were placed in an oven at 500 °C for 1.5 h, and the test material was left to cool in an isolated place.

Calculations:

1 mg barium sulfate precipitation: 0.137 mg sulfur or 0.343 SO_3_

Sulfate in ammonium nitrate:

(2) S,%=W×0.137×(V1V2)×M

(3) $${\text{SO}}_{3},\text{\%}=\text{S},\text{\%}\times 2.5$$

where W is the mass of barium sulfate in precipitation, V_1_ is the sample volume, V_2_ is the total volume, M is the sample mass.

### 2.6 Analysis of silicic acid

The chemicals used were diluted HCl (50%), sulfuric acid (98%), and hydrofluoric acid (48%). The sample that contained silicate (0.25 g) was added to a platinum cup, heated, and placed for 1 h in an oven at 500 °C. The sample was mixed with 10 mL HCl (50%, w/w) and diluted with demineralized water to 100 mL. The water was then fully vaporised in a water bath, followed by the addition of 8–10 drops HCl and 50 mL water. This solution was covered with a watch glass and then filtered through Whatman filter paper No. 42. The filter paper was placed in a platinum cup and 2–3 drops of concentrated sulfuric acid were added. This paper was heated at 1000 °C for 0.5 h in an ash furnace, then cooled and weighed, followed by the addition of 2 drops of sulfuric acid. After this, HF (48%, w/w) was added to 25 mL of the original volume. Silicon fluoride was vaporised at 250 °C for 1 h in a traditional oven. This solution was kept at 1000 °C for 0.5 h in an ash furnace then cooled and weighed.

Calculations:

(4) SiO2,mgL−1=(weightloss×100)sampleamount,mL

### 2.7 Analysis of nitrogen

Approximately 7 g of a nitrogenous fertiliser sample was used for the analysis. The sample was diluted with demineralized water to 500 mL. Then, 10 mL of this solution was withdrawn and mixed with 50 mL of 20% NaOH. The resulting mixture was titrated against standard sulfuric acid (98%, w/w).

The article "A novel industrial-scale strategy to prevent degradation and caking of ammonium nitrate" was published in 2020. Journal: Heliyon.

Calculations:

(5) N,%=(50−A)×F

where A is the volume of NaOH during titration and F is the dilution factor.

### 2.8 XRD analysis of calcium lignosulfonate in ammonium nitrate

Calcium lignosulfonate were subjected to mineralogical analysis using X-ray diffraction (XRD) with a PANalytical V4.1 instrument, utilizing the Rietveld-based X'Pert HighScore Plus software to identify and semi-quantify minerals [25].

## 3 Results and discussion

The experiments carried out in this study were carried out in the Toros Agri&Industry (Mersin, Turkey) R&D center and ammonium nitrate production was carried out under operating conditions in the ammonium nitrate production facility of the same factory.

There are various approaches to chemicals used in the literature. Various references are provided in the references on the use of these resources [4]. With similar approaches, it was decided which concentrations to use. However, the relative humidity of the air in the storage conditions of the produced ammonium nitrate (Mersin, Turkey) varies between 45-89% and the temperature in the range of 25–39 °C.

Ammonium nitrate fertiliser is obtained by the reaction between nitric acid (55%, w/w) and anhydrous ammonia during ammonium nitrate production, as per the EFMA. According to commercial patents [14], several methods were used during production, and investigations were performed to realise production at the lowest cost and dilution rate, according to the producer's requirements. Ammonium nitrate production includes reaction stages with several inputs and parameters. First, anhydrous ammonia is vaporised (22 °C, 5.6 kg/cm^2^) with oxygen for obtaining nitric oxide, which is then reacted with air to obtain nitrogen oxide and thus, nitric acid is produced. Nitric acid is then reacted with anhydrous ammonia to produce ammonium nitrate salt [26].

The related method is shown by EFMA [26] among the standard ammonium nitrate production methods and there are facilities producing with the same method. There are several studies reported in the literature about the reactions of chemicals applied in the method with ammonium nitrate.

In the vacuum concentrating method in the first stage, the 80% concentration of ammonium nitrate produced is based on the principle of concentrating to 99.7% concentration by two-stage evaporation. It is based on the principle of removing the water vapor released as a result of evaporation in the first stage in vacuum reaction medium, concentrating from 80% concentration to 94%, and applying the same method for the second time to concentrate the 94% concentration of ammonium nitrate to 99.7% concentration [26].

The article "A novel industrial-scale strategy to prevent degradation and caking of ammonium nitrate" was published in 2020. Journal: Heliyon.

According to consumer requirements, ammonium nitrate can be produced with 26% or 33% nitrogen and as pure ammonium nitrate. This nitrogen content is obtained by using chemicals such as a calcium carbonate addition in the dilution stage. For obtaining 26% nitrogen content, 250 kg of calcium carbonate is added to 1000 tons of ammonium nitrate, and for obtaining 33% nitrogen content, 60 kg of calcium carbonate is added [17]. In this study, sodium silicate is added to minimise the amount of CO_2_ created from calcium carbonate added at the dilution stage. Due to cost factors, sodium silicate is added at 50% concentration with respect to calcium carbonate. Another chemical added to minimise CO_2_ gas formation is 600 ppm sulfuric with nitric acid. To overcome the double salt problem, silicic acid is added at the dilution stage. In the prilling stage, a prilling bucket that rotates at 150–300 rpm is used. The rotation speed of the prilling bucket affects the particle size. The average particle size is 2 mm, which is considered the standard value by EFMA.

Chemical additives are added to decrease agglomeration and caking to the fertiliser solution that is concentrated to 99.7%. For diluting ammonium nitrate, calcium carbonate is the most widely used. Sodium silicate is another chemical that can be added for diluting. In ammonium nitrate production, reactions between carbonate and silicate must be monitored. In this study, because of the addition of sodium silicate, no gas output or foaming reaction was observed.

Another chemical used for investigating the behaviour of fertiliser particles is silicic acid. Many studies have been carried out to elucidate the effects of silicic acid on fertiliser production [14]. Silicic acid is added to eliminate sulfuric acid, which leads to the formation of double salts with nitrate in ammonium nitrate.

When calcium carbonate is added to an ammonium nitrate solution, CO_2_ is created. This causes a foaming reaction. To prevent the foaming reaction, sulfuric acid has been added to the ammonium nitrate solution. It was expected that the sulfate resulting from the addition of sulfuric acid to the solution, would form CaSO_4_ and NH_4_SO_4_, but the amount of sulfuric acid added was too low (600 ppm) and the presence of sulfate salts such as the CaSO_4_ and NH_4_SO_4_ continued to cause the foaming reaction [1]. However, after ammonium nitrate production, these sulfate salts caused the creation of a sulfate-nitrate double salt [4]. Therefore, creation of possible sulfate-nitrate double salts has been minimised by adding silicic acid, which eliminates sulfate salts in the reaction (Figure 2).

The article "A novel industrial-scale strategy to prevent degradation and caking of ammonium nitrate" was published in 2020. Journal: Heliyon.

**Figure 2:** (a) Ion chromatogram for ammonium nitrate that contains only calcium carbonate; (b) ion chromatogram for ammonium nitrate that contains calcium carbonate, sodium silicate, and silicic acid.

In terms of reproducibility of the results, two separate trials were made in all analysis methods for each sample and no problems were observed at the point of compliance with the production conditions.

Sulfuric acid is added to the fertiliser solution to consume CO_2_ that is formed by the addition of calcium carbonate. SEM images (Figures 3, 4, and 5) and sieve analysis (Tables 1 and 2) show that degradation is suppressed by the addition of silicic acid, and the agglomeration of ammonium nitrate is prevented.

**Figure 3:** (a) SEM images of ammonium nitrate that contains calcium carbonate (25%); (b) SEM images of ammonium nitrate containing calcium carbonate (12.5%) and sodium silicate (12.5%).

**Figure 4:** (a) SEM image of ammonium nitrate that contains silicic acid (1 mL silicic acid/5.6 mL sulfuric acid), calcium carbonate (12.5%), and sodium silicate (12.5%); (b) SEM image of ammonium nitrate that contains calcium carbonate (25%) after a two-year storage period.

**Figure 5:** (a) SEM image of ammonium nitrate that contains calcium carbonate (12.5%) and sodium silicate (12.5%) after two years of storage; (b) SEM image of ammonium nitrate that contains silicic acid (1 mL silicic acid/5.6 mL sulfuric acid), calcium carbonate (12.5%), and sodium silicate (12.5%) after a two-year storage period.

**Table 2:** Screen sieve, crushing strength and chemical composition analyses for ammonium nitrate containing only calcium carbonate, freshly produced and at the end of the two-year storage. The averages for multiple samples are presented.

Period (month)	3.35 mm	2.5 mm	2.0 mm	1.0 mm	0.5 mm	U.S. (mm)	Crushing Strength	${\text{SO}}_{4}^{2-}$	N (%)
Trial 1									

Final product	2.5	41.6	35.3	19.2	1.4	0	2.52	6.51	26.33
Final product after two years	5.0	44.2	36.2	12.9	1.7	0	1.82	6.40	25.92

Trial 2									

Final product	2.4	41.7	35.4	19.1	1.4	0	2.57	6.53	26.41
Final product after two years	5.2	44.3	36.4	12.7	1.4	0	1.86	6.43	25.89

According to SEM images (Figure 3 (a)), the cracking is not found on the surface of ammonium nitrate that contains CaCO_3_. Conversely, according to Figure 3(b), cracking was found on the surface of ammonium nitrate in the presence of sodium silicate due to a decrease in surface tension on the surface of the ammonium nitrate. According to SEM images (Figure 4 (a)), it has been observed that the addition of silicic acid increases the surface tension of ammonium nitrate that contains CaCO_3_ and sodium silicate, which decreases surface cracking (Figure 3(b)). Deformation was seen due to bulk pressure in the samples of ammonium nitrate. At the end of two years in storage, the surface of the ammonium nitrate contained CaCO_3_ (Figure 4(b)). The effect of sodium silicate and silicic acid additions on the crushing strength of ammonium nitrate particles is shown in Figure 5 (a, b). The figure shows the effect of bulk pressure on ammonium nitrate, along with sodium silicate additions to ammonium nitrate, which saves the ammonium nitrate according to the addition of CaCO_3_. Furthermore, at the end of two years in storage, and because the addition of silicic acid to ammonium nitrate solution prevents creation of sulfate-nitrate double salt, surface tension had decreased. This result is seen as less surface deformation in Figure 5(b).

The article "A novel industrial-scale strategy to prevent degradation and caking of ammonium nitrate" was published in 2020. Journal: Heliyon.

When SEM images (Figures 3, 4, and 5) are examined, it is seen how each additive affects the crystal structure. According to this analysis, the crystal structure has reached a more stable structure with the addition of sodium silicate (Figure 3b) and contributed to the acceleration of the phase transformation by responding to the cooling process faster within the prilling tower.

On the other hand, it is observed that silicic acid additive (Figures 4a, 5b) strengthens the crystal structure and thus decreases the tendency to degradation since it minimizes the sulfate-derived double salt formation.

In this respect, it can be said that for the purpose of dilution, the final product temperature is more stable with the addition of sodium silicate (Figures 3b, 4a, 5a, 5b) and silicic acid (Figures 4a, 5b) with the addition of sodium silicate (Figures 3b, 4a, 5a, 5b) and silicic acid (Figures 4a, 5b) compared to the ammonium nitate production processes in which calcium carbonate is used alone. Calcium lignosulfonate salt is another phenomenon observed in the cooling process, in which the ammonium nitrate increases the cooling rate and affects the crystal structure of ammonium nitrate, completing the phase conversion.

This study is novel in that ion chromatography, electron microscopy, and screen sieve analyses of ammonium nitrate are conducted on an industrial scale product. It is difficult to store the produced ammonium nitrate because it is a strong oxidant and is hygroscopic. This is related to the phase change of ammonium nitrate, so degradation can be prevented by the addition of chemicals such as sodium silicate. This compound can be mixed with calcium chloride to precipitate calcium silicate [21], which is widely used in the nitrogenous fertiliser industry [1]. This increases the amount of calcium silicate in the soil that did not contain it previously. In this study, a better chemical composition than that in several patented chemicals is suggested to prevent the degradation of ammonium nitrate crystals.

The article "A novel industrial-scale strategy to prevent degradation and caking of ammonium nitrate" was published in 2020. Journal: Heliyon.

The results of sieve analysis show that the particle size of ammonium nitrate containing calcium carbonate is smaller than that of ammonium nitrate containing sodium silicate during production. The particle size increases with the addition of both sodium silicate and calcium carbonate (Table 3), as opposed to the case of addition of calcium carbonate only (Table 2). Thus, better results were obtained with the mixture of sodium silicate and calcium carbonate for mitigating the degradation problem. The resulting CO_2_ causes foaming on the surface of the ammonium nitrate solution. This in turn leads to deformation of ammonium nitrate prills during the addition of calcium carbonate.

**Table 3:** Screen sieve, crushing strength and chemical composition analyses for ammonium nitrate containing calcium carbonate (12.5%), sodium silicate (12.5%), and silicic acid (1 mL silicic acid/5.6 mL sulfuric acid), freshly produced and at the end of the two-year storage. The averages for multiple samples are presented.

Period (month)	3.35 mm	2.5 mm	2.0 mm	1.0 mm	0.5 mm	U.S. (mm)	Crushing Strength	${\text{SO}}_{4}^{2-}$	N (%)	SiO_2_ (ppm)
Trial 1										

Final product	6.9	48.7	41.2	2.7	0.5	0	2.42	1.11	26.55	0.175
Final product after two years	8.5	48.4	38.8	3.4	0.9	0	2.29	0.91	26.01	0.169

Trial 2										

Final product	6.8	48.5	41.5	2.6	0.6	0	2.45	1.13	26.45	0.181
Final product after two years	8.3	48.9	38.5	3.1	1,2	0	2.23	0.95	26.21	0.172

To suppress the foaming reaction, the amount of CO_2_ should be decreased [1]. In various patented studies, sulfuric acid is added to the reaction ambience in order to prevent the formation of CO_2_ during ammonium nitrate production. Sulfuric acid can lead to the formation of double salts such as sulfate-nitrate after production, depending on the storage conditions. The double salt creates crystal bridges for accelerating the degradation of ammonium nitrate. These crystal bridges cause breaking between the particles by weakening the hydrogen bonds. To minimize the amount of sulfate, silicic acid was used to eliminate sulfuric acid during the production process. It was found that 1 mL silicic acid eliminated 5.6 mL sulfuric acid. SEM images showed that the extent of degradation of ammonium nitrate that contains sodium silicate is lower than that of ammonium nitrate containing calcium carbonate. During two years of storage under 0.28 kg/cm^2^ pressure, the surface of ammonium nitrate that contains sodium silicate is deformed to a greater extent than that of ammonium nitrate containing calcium carbonate (Figures 4 (b) and 5 (b)).

The article "A novel industrial-scale strategy to prevent degradation and caking of ammonium nitrate" was published in 2020. Journal: Heliyon.

The SEM images in Figures 3 (a) and 4 (b) show the surface of ammonium nitrate that contains only calcium carbonate. Figures 3 (b) and 5 (a) reveal the surface morphology of ammonium nitrate containing both calcium carbonate (12.5%) and sodium silicate (12.5%).

Furthermore, silicic acid eliminates the double salts (Figures 4 (a) and 5 (b)). According to these investigations, the best surface properties are obtained by the addition of sodium silicate, calcium carbonate, and silicic acid. When sodium silicate and calcium carbonate are added to the reaction ambience, the crushing strength of ammonium nitrate is higher (Table 3) than that of ammonium nitrate to which only calcium carbonate is added (Table 2). Ion chromatography is used to investigate the ammonium nitrate degradation progress. The main purpose here is to observe the effects of silicic acid on the sulfate salts.

In the present study, the sulfate content in ammonium nitrate was found to decrease after a two-year storage period. The amount of sulfate ions was found to be quite low during this storage period because silicic acid was added to the reaction ambience to eliminate the sulfuric acid during ammonium nitrate production (Figure 2 (a), (b)). Ion chromatography analysis was conducted for ammonium nitrate that contains only calcium carbonate and for that containing sodium silicate (12.5%), calcium carbonate (12.5%), and silicic acid (1 mL silicic acid/5,6 mL sulfuric acid). This analysis was not conducted for ammonium nitrate containing calcium carbonate and sodium silicate because sodium silicate is an inorganic material that does not cause the foaming reaction to form CO_2_. CO_2_ production is only seen in the reaction between calcium carbonate and sodium silicate. In this case, sulfuric acid and silicic acid are not used.

In this study, lignosulfonate was added for linking the crystals of ammonium nitrate to one another during the prilling process. Therefore, lignosulfonate salts are expected to lose their chemical structure during the two-year storage period. The XRD analysis showed that the concentration of lignosulfonate in ammonium nitrate does not change in the ammonium nitrate fertiliser (Figure 6). Moreover, lignosulfonate acts as a filler material for the porous structure on the surface of ammonium nitrate that contains calcium carbonate, sodium silicate, and silicic acid.

**Figure 6:** XRD diffractograms of calcium lignosulfonate in ammonium nitrate during the two-year storage period with varying calcium lignosulfonate (wt%).

The article "A novel industrial-scale strategy to prevent degradation and caking of ammonium nitrate" was published in 2020. Journal: Heliyon.

XRD results for the calcium lignosulfonate during ammonium nitrate storage in Figure 6. The XRD analysis was used to determine the lignosulfonate content in the Ammonium nitrate. As expected, the two samples analysed have low values (0.027–0.030%)

The said amounts of silicic acid, sodium silicate and calcium carbonate are the optimum values obtained in the research study. For example, the addition of sodium silicate, the cooling solidified ammonium nitrate pore structure and crushing strength was maximised. Silicic acid was added to minimise the foaming reaction of sulfuric acid in the presence of CO_2_ while not completely destroying the effect of sulfuric acid in the environment. Silicic acid is introduced into the ammonium nitrate reaction ambience in order to eliminate excess sulfuric acid remaining as a result of the foaming reaction.

With the addition of chemicals used to complete the phase transformation, ammonium nitrate, by entering a rapid solidification process showed reduced caking tendency in storage for two years; moreover, its hygroscopic properties and moisture content decreased during production.

In previous studies [1, 2, 4], degradation and caking of ammonium nitrate has been reported; if it absorbs moisture before it cakes, it degrades, resulting in the loss of its physical and chemical properties. Thus, in order to prevent a caking, sodium silicate, added to the reaction mixture, has a hardening effect, that is, crushing strength is increased and the pore structure is reduced. Thus far, in the ammonium nitrate production process, solidification of this compound with the addition of calcium lignosulfonate to effect phase conversion in the solidification process has not been reported in the literature. Herein, the solution of caking and degradation problems of ammonium nitrate are addressed. In this respect, methodology of ammonium nitrate production proposed in this study will provide an important alternative to the manufacturers in terms of troubleshooting during as the synthesis of this compound.

In addition to these, the use of sodium silicate added in the reaction medium in combination with calcium carbonate will not add an additional cost to the process, due to the intense supplier potential and easy access, in the research conducted on the process structure and the selection of the cheapest chemicals possible due to the solution of the problem. Because the calcium carbonate used for dilution has the same price properties.

On the other hand, although the number of suppliers is quite low in nature, silicic acid will not create a big load for the process, since less than 20% of sulfuric acid (600 ppm) is used as a chemical additive. Calcium lignosulfonate, on the other hand, is an easily accessible chemical due to its intensive use of binders in many industrial establishments such as cement, and because of its extensive supplier network, it will affect the cost of a typical ammonium nitrate production process by 1%, since it is used in the proposed process at a rate of 0.5%.

The article "A novel industrial-scale strategy to prevent degradation and caking of ammonium nitrate" was published in 2020. Journal: Heliyon.

According to the EFMA (European Fertilizer Manufacture Association) standards, after the production of ammonium nitrate fertilizer, it should not show any degradation reaction in the 2-year storage period. In the chemical addition and methods previously reported in the literature, the 2-year storage period of ammonium nitrate cannot be guaranteed. With the method proposed in this study, no significant change in the physical and chemical structure of ammonium nitrate was observed over a 2-year period.

The use of sodium silicate added in the reaction medium in combination with calcium carbonate will not add an additional cost to the process, due to the intense supplier potential and easy access, in the research conducted on the process structure and the selection of the cheapest chemicals possible due to the solution of the problem. Because the calcium carbonate used for dilution has the same price properties.

On the other hand, although the number of suppliers is quite low in nature, silicic acid will not create a big load for the process, since less than 20% of sulfuric acid (600 ppm) is used as a chemical additive. Calcium lignosulfonate, on the other hand, is an easily accessible chemical due to its intensive use of binders in many industrial establishments such as cement, and because of its extensive supplier network, it will affect the cost of a typical ammonium nitrate production process by 1%, since it is used in the proposed process at a rate of 0.5%.

## 4 Conclusions

In this study, it was studied to add chemicals such as calcium carbonate, sodium silicate, silicic acid and calcium lignosulfonate to the production process to prevent the high moisture absorption potential of ammonium nitrate. The applied ammonium nitrate production method is a two-stage ammonium nitrate production process. No degradation was observed in the structure of ammonium nitrate particles produced by this production method during the 2-year storage period. In this respect, it is longer lasting than ammonium nitrate particles produced by the production methods reported so far in the literature.

Along with chemical analyses, the nitrogen value of the ammonium nitrate fertilizer produced does not lose its initial value significantly within the specified time period, can be seen as a commercially important development. However, all chemicals used are easily accessible in the production of ammonium nitrate and can be offered to the manufacturer as an important alternative for the solution of the problem, since it has a low commercial value and does not affect the process cost by more than 1%.

The article "A novel industrial-scale strategy to prevent degradation and caking of ammonium nitrate" was published in 2020. Journal: Heliyon.

Sodium silicate is a good alternative to calcium carbonate, which is used for the dilution of ammonium nitrate during production, and silicic acid fully eliminates sulfate ions in ammonium nitrate. Thus, silicic acid prevents the creation of double salts in ammonium nitrate, and the optimal concentration of calcium lignosulfonate used as a binding material for ammonium nitrate particles in the prilling process is determined as 0.5%. Hence, calcium lignosulfonate is supplied to improve the crushing strength of ammonium nitrate. At the end of two years of storage, there is a negligible loss of nitrogen content with the addition of the aforesaid chemicals. According to these results, the chemical compositions and methods employed in this study are feasible for ammonium nitrate fertiliser manufacturers.

In the ammonium nitrate production methods applied to date, the effects of chemicals added either by coating form or as chemical additive to the process had a lifetime of less than 6 months. In order to increase the 2-year storage process as a standard in the fertilizer industry, none of these methods showed the desired performance and showed a tendency to degrade over a period of 6 months. No degradation was observed in the ammonium nitrate particles produced in its standard form in the 2-year time period with the method applied in this study.

## Declarations

### Author contribution statement

Ahmet Ozan Gezerman: Conceived and designed the experiments; Performed the experiments; Analyzed and interpreted the data; Contributed reagents, materials, analysis tools or data; Wrote the paper.

### Funding statement

This research did not receive any specific grant from funding agencies in the public, commercial, or not-for-profit sectors.

### Competing interest statement

The authors declare no conflict of interest.

### Additional information

No additional information is available for this paper.
